# Ultra-short-term heart rate variability during resistance exercise in the elderly

**DOI:** 10.1590/1414-431X20186962

**Published:** 2018-05-21

**Authors:** G.P.T. Arêas, F.C.R. Caruso, R.P. Simões, V. Castello-Simões, R.B. Jaenisch, T.O. Sato, R. Cabiddu, R. Mendes, R. Arena, A. Borghi-Silva

**Affiliations:** 1 Departamento de Ciências Fisiológicas, Instituto de Ciências Biológicas, Universidade Federal do Amazonas, Manaus, AM, Brasil; 2 Departamento de Fisioterapia, Pós Graduação em Fisioterapia, Universidade Federal de São Carlos, São Carlos, SP, Brasil; 3 Departamento de Fisioterapia, Curso de Fisioterapia, Universidade Federal de Santa Maria, Santa Maria, RS, Brasil; 4 Department of Physical Therapy, College of Applied Health Sciences, University of Illinois Chicago, Chicago, IL, USA

**Keywords:** Autonomic function, Older people, Leg press

## Abstract

Despite the appeal of ultra-short-term heart rate variability (HRV) methods of analysis applied in the clinical and research settings, the number of studies that have investigated HRV by analyzing R-R interval (RRi) recordings shorter than 5 min is still limited. Moreover, ultra-short-term HRV analysis has not been extensively validated during exercise and, currently, no indications exist for its applicability during resistance exercise. The aim of the present study was to compare ultra-short-term HRV analysis with standard short-term HRV analysis during low-intensity, dynamic, lower limb resistance exercise in healthy elderly subjects. Heart rate (HR) and RRi signals were collected from 9 healthy elderly men during discontinuous incremental resistance exercise consisting of 4-min intervals at low intensities (10, 20, 30, and 35% of 1-repetition maximum). The original RRi signals were segmented into 1-, 2-, and 3-min sections. HRV was analyzed in the time domain (root mean square of the of differences between adjacent RRi, divided by the number of RRi, minus one [RMSSD]), RRi mean value and standard deviation [SDNN] (percentage of differences between adjacent NN intervals that are greater than 50 ms [pNN50]), and by non-linear analysis (short-term RRi standard deviation [SD1] and long-term RRi standard deviation [SD2]). No significant difference was found at any exercise intensity between the results of ultra-short-term HRV analysis and the results of standard short-term HRV analysis. Furthermore, we observed excellent (0.70 to 0.89) to near-perfect (0.90 to 1.00) concordance between linear and non-linear parameters calculated over 1- and 2-min signal sections and parameters calculated over 3-min signal sections. Ultra-short-term HRV analysis appears to be a reliable surrogate of standard short-term HRV analysis during resistance exercise in healthy elderly subjects.

## Introduction

Heart rate variability (HRV) analysis provides a quantification of heart rate (HR) and beat-to-beat fluctuations, and is the most frequently used approach to assess cardiac autonomic balance (1). HRV analysis is a simple, inexpensive, and well-validated tool that provides, among others, significant prognosis markers for coronary heart disease (2), cardiac (3) and all-cause mortality, all of which can be calculated in resting conditions (4). HRV indices have been used to assess the autonomic HR control in physiological conditions, including exercise for adult and elderly subjects (5 [Bibr B06] [Bibr B07]–8). Furthermore, studies show that HRV analysis is an important tool for exercise prescription and for the evaluation of adaptations to exercise training (9).

Recent studies evaluated the autonomic nervous HR control during steady-state aerobic exercise (10) and during dynamic resistance exercise, including upper- and lower-limb exercise in elderly subjects (10–13). Simões et al. (10) analyzed the cardiac autonomic response during dynamic resistance exercise in elderly men and showed high correlation and concordance between lactate threshold and cardiac autonomic behavior. However, their protocol included prolonged exercise duration (4 min), with approximately 48 repetitions for each series of exercise, which is not recommended in clinical practice, according to the American College of Sports Medicine (ACSM) (14).

Recently, ultra-short-term HRV analysis has been proposed as an alternative approach to assess autonomic balance. Previous studies have shown that ultra-short-term HRV analysis could be performed on HRV signals shorter than 5 min during rest (15–22) as well as before and after physical activity (23,24). However, to our knowledge, no studies have analyzed the autonomic modulation of HR by ultra-short-term HRV analysis during resistance exercise in healthy elderly subjects. Considering that low intensities and repetitions of resistance exercise are normally recommended for this population, ultra-short-term HRV analysis could represent an important tool for the evaluation of autonomic control during this exercise modality.

Thus, the aim of the present study was to assess the application of ultra-short-term HRV analysis during low-intensity, dynamic resistance exercise in healthy elderly subjects, using a 45° leg press. We hypothesized that HRV indices obtained over ultra-short time series (1- and 2-min stationary signal sections) would be similar to those obtained over standard duration time series (3-min stationary signal sections) selected from the signals recorded during the whole exercise session (4 min).

## Material and Methods

### Study protocol

Nine healthy male volunteers (age, 65±3) were recruited to participate in the present study. Following anamnesis, volunteers were familiarized with the experimental equipment and procedures. All study objectives, experimental procedures, and risks were described in detail, and subjects signed a written informed consent form before initiation of the study. The Ethics Committee for Human Research of the Universidade Federal de São Carlos, São Carlos, SP, Brazil, approved the investigation. Subjects were excluded if they presented cardiovascular problems, were current smokers, were taking any type of medication, had participated in a regular exercise program in the 6 months preceding the study, presented musculoskeletal pain, or had difficulty in understanding or completing the exercise protocol. All subjects were evaluated in the morning to avoid differing physiological responses due to circadian changes.

The experiments were carried out over a period of 2 days, 1 week apart, in a climatically controlled room at 22–24°C, with relative air humidity at 50–60%. The day before data collection, subjects were taken to the experimental room for familiarization with the procedures and equipment to be used. All subjects were instructed to avoid caffeinated and alcoholic beverages or any other stimulants the night before and the day of data collection. They were also instructed not to perform activities requiring moderate-to-heavy physical exertion the day before data collection. Lastly, subjects were instructed to avoid heavy meals 2 h before the tests. Immediately before data collection, subjects were interviewed and examined to confirm their good health status, the occurrence of a normal night's sleep, and that HR and systemic blood pressure (BP) were within the normal range. The volunteers were instructed to avoid speaking unnecessarily before, during, and after exercise.

### 1-repetition maximum test (1-RM)

The 1-RM test was performed by gradually increasing resistance until the volunteer succeeded in performing no more than 1 repetition on a 45° leg press (Pró-Fitness, São Paulo, SP, Brazil) (25). During the test, the volunteer maintained a seated position on the equipment with the trunk inclined at 45° from the ground, with the knees and hips flexed at 90°. During the movement, the knees and hips were extended and returned to their initial position. Before the execution of the test, subjects were oriented to avoid isometric contraction and exhale during the extension of the knees and hips to avoid the Valsalva maneuver (26). The resistance load for 1-RM was estimated (1-RM-E) before the test by multiplying the volunteer's body weight by 4, based on a previous study (11 [Bibr B12]).

The initial resistance load applied to determine 1-RM was 80% 1-RM-E, and if the subject was able to perform more than 1 complete movement, the load was increased by 10% 1-RM-E after a 5-min rest interval between trials. When the first attempt was unsuccessful because the resistance load had been overestimated, the load was reduced by 10% 1-RM-E. Once the pre-training 1-RM was determined, a second attempt with an additional 10% was performed to verify the load value. If the individual was not successful on this second attempt, the previous load was considered as their 1-RM. However, if the subject was successful, a new load was added until 1-RM was determined. Based on the 1-RM-E loads, it was expected that 1-RM would be determined within 6 attempts (27).

### Discontinuous incremental exercise

The exercise protocol was done 1 week after the 1-RM test. After a 10-min rest on the equipment, the discontinuous incremental exercise protocol was initiated at a load of 10% 1-RM, with 10% 1-RM increases until reaching a load of 30% 1-RM, and subsequent 5% 1-RM increases until exhaustion. At each different percentage, the volunteer performed 4 min of exercise at a movement rhythm of 12 repetitions per minute, maintaining respiratory cadence, with each repetition performed in 5 s (2 s of knee and hip extension and 3 s of flexion). The electrocardiographic (ECG) activity was monitored and the RRi signal was collected by a Polar S810i heart rate monitor (Polar, Finland), while the movement rhythm was controlled by verbal commands. The recovery period between trials was 15 min. Before, during, and after the exercise protocol, ECG and BP were monitored. Lower limb fatigue and muscle pain were assessed by the modified Borg Scale (28) at the end of each maneuver. Termination criteria for the exercise protocol were as follows: 1) incapacity of the subject to perform the movement with proper form; 2) excessive increase in systolic BP (SBP; i.e., >200 mmHg); 3) reaching 85% of maximum HR [(220-age) × 0.85]; 4) ECG abnormalities, or 5) voluntary exhaustion.

### HRV measures

The RRi signal was collected by a Polar S810i heart rate monitor; the time series were verified and corrected using a detection algorithm followed by a visual inspection. The RRi time series were resampled at 5 Hz by equidistant linear interpolation. Signals were filtered in order to remove oscillations below 0.04 Hz and over 1.0 Hz. For each 4-min signal portion recorded during resistance exercise, the most stable 3-min portion was selected. The initial 40 seconds of recording were discarded (1). Afterwards, three different signal portions were considered for each signal: the first 1-min signal portion, the first 2-min signal portion, and the whole 3-min signal, as shown in Figure 1.

**Figure 1.** Illustration of a heart rate variability signal acquired during dynamic resistance exercise at an intensity of 30% 1-repetition maximum test and its subdivision in 1-, 2-, and 3-min portions. RR: time between R waves.

HRV indices were analyzed using Kubios HRV Analysis Software 2.0 for Windows (The Biomedical Signal and Medical Imaging Analysis Group, Department of Applied Physics, University of Kuopio, Finland). Time domain HRV indices included: i) HR_mean_; ii) the square root of the mean of the sum of the squares of differences between adjacent RRi, divided by the number of RRi minus 1 (RMSSD) [1]; iii) the RRi mean value and standard deviation (SDNN); and iv) percentage of differences between adjacent NN intervals that are greater than 50 ms (pNN50). A non-linear analysis was performed, consisting of the computation of the Poincaré plot descriptors SD1 and SD2. Specifically, SD1 represents the dispersion of points perpendicular to the line of identity and provides information about the instantaneous beat-to-beat variability; SD2 represents the RRi long-term standard deviation and is considered a parasympathetic and sympathetic modulation marker.

### Statistical analysis

Data are reported as means±SD. Data distribution was verified by the Shapiro-Wilk test. To analyze the difference between indices obtained from tachogram portions of different duration, one-way analysis of variance (ANOVA) for repeated measurements with *post hoc* Bonferroni test was used. To analyze the concordance between 1- and 2-min signal portions and 3-min signals, the intraclass correlation coefficient (ICC) was computed. Values between 0 and 0.30 were considered small, values between 0.31 and 0.49 were considered moderate, values between 0.50 and 0.69 were considered large, values between 0.70 and 0.89 were considered excellent, and values between 0.90 and 1.00 were considered near perfect (29). In addition, Bland-Altman plots were used to identify the upper and lower limits of agreement of RMSSD and SD1 between 3- and 2-min signals and between 3- and 1-min signals at different resistance exercise loads (30). The analysis was performed using SPSS software 17.0 (SPSS IMB, USA) and GraphPad prism 5.0 (GraphPad, USA). P<0.05 was considered statistically significant for all tests.

## Results

All volunteers successfully completed the incremental resistance exercise protocol without any complaints. The maximal load achieved was 35% of 1-RM in all volunteers, with 4 min of uninterrupted resistance exercise.

The volunteers' anthropometric and clinical characteristics are summarized in Table 1. Table 2 shows the time domain and non-linear HRV indices obtained at different exercise intensities from 3-, 2-, and 1-min tachogram sections. No statistical difference was found between time series of different duration (3, 2, and 1 min) for any of the studied parameters (P<0.05). Table 3 shows that excellent to near-perfect association was observed at all exercise loads between linear and non-linear parameters calculated over 1- and 2-min signals and parameters calculated over 3-min signals.

**Table 1.** Anthropometric and clinical characteristics of the study population.

Characteristics	n=9
Age (years)	65±3
Height (m)	1.7±0.2
Weight (kg)	69±7
BMI (m/kg^2^)	24±2
HR rest (bpm)	62±9
SBP rest (mmHg)	124±7
DBP rest (mmHg)	79±4

Data are reported as means±SD. BMI: body mass index; HR: heart rate; SBP: systolic blood pressure; DBP: diastolic blood pressure.

**Table 2.** Average linear and non-linear heart rate variability parameters calculated over 3, 2, and 1 min signals recorded at different exercise intensities.

	3 min	2 min	1 min	P value
Time Domain				
R-Ri (ms)				
10% 1-RM	819±93	813±92	804±91	0.9
20% 1-RM	787±107	788±105	788±107	1.0
30% 1-RM	759±94	765±96	770±98	0.9
35% 1-RM	732±89	744±94	752±98	0.9
SDNN (ms)				
10% 1-RM	31±13	32±13	33±13	0.9
20% 1-RM	26±8	27±8	25±9	0.8
30% 1-RM	23±10	24±11	22±12	0.9
35% 1-RM	20±7	21±8	21±8	0.9
rMSSD (ms)				
10% 1-RM	27±16	27±15	27±15	0.9
20% 1-RM	20±10	20±9	19±10	0.9
30% 1-RM	18±8	19±9	18±12	0.9
35% 1RM	17±9	17±9	17±11	0.9
pNN50 (%)				
10% 1-RM	9±13	11±16	12±14	0.9
20% 1-RM	4.9±7.6	5.3±7.6	5.0±7.7	0.9
30% 1-RM	2.8±4.1	3.6±5.1	4.6±8.3	0.8
35% 1-RM	3.0±5.0	3.2±5.0	4.7±6.9	0.8
Non-linear Domain				
SD1 (ms)				
10% 1-RM	19±11	19±11	19±10	0.9
20% 1-RM	14±7	14±6	14±7	0.9
30% 1-RM	12±6	13±6	13±8	0.9
35% 1-RM	12±6	12±6	13±8	0.9
SD2 (ms)				
10% 1-RM	54±31	56±30	48±19	0.8
20% 1-RM	39±11	41±11	39±13	0.9
30% 1-RM	41±13	41±13	39±15	0.9
35% 1-RM	45±13	38±13	32±13	0.1

Data are reported as means±SD. RRi: RR intervals mean value; SDNN: RR intervals standard deviation; RMSSD: root mean square of the successive differences between adjacent RRi, divided by the number of RRi minus one; pNN50: percentage of differences between adjacent NN intervals that are greater than 50 ms; SD1: standard deviation type I; SD2: standard deviation type II. 1-RM: 1-repetition maximum test. ANOVA with *post hoc* Bonferroni test was applied.

**Table 3.** Intraclass correlation coefficient (ICC) between linear and non-linear parameters calculated at different exercise intensities over 1 and 2 min signals and parameters calculated over 3 min signals.

	10% 1-RM		20% 1-RM		30% 1-RM		35% 1-RM	
	1 min	2 min	1 min	2 min	1 min	2 min	1 min	2 min
Time domain								
HR_mean_ (1/min)	0.975	0.819	0.999	1.000	0.995	0.999	0.998	0.995
	(0.0001)	(0.02)	(0.0001)	(0.0001)	(0.0001)	(0.0001)	(0.0001)	(0.0001)
RRi (ms)	0.996	0.882	1.000	1.000	0.998	0.994	0.984	0.994
	(0.0001)	(0.0006)	(0.0001)	(0.0001)	(0.0001)	(0.0001)	(0.0001)	(0.0001)
SDNN (ms)	0.990	0.784	0.937	0.991	0.921	0.992	0.967	0.996
	(0.0001)	(0.03)	(0.0001)	(0.0001)	(0.001)	(0.0001)	(0.0001)	(0.0001)
RMSSD (ms)	0.961	0.946	0.968	0.994	0.919	0.987	0.972	0.996
	(0.0002)	(0.0001)	(0.0001)	(0.0001)	(0.002)	(0.0001)	(0.0001)	(0.0001)
pNN50 (%)	0.961	0.952	0.989	0.997	0.827	0.974	0.948	0.985
	(0.0001)	(0.0001)	(0.0001)	(0.0001)	(0.011)	(0.0001)	(0.0001)	(0.0001)
Non-linear domain								
SD1 (ms)	0.962	0.947	0.83	0.831	0.917	0.986	0.917	0.982
	(0.0001)	(0.0001)	(0.008)	(0.014)	(0.001)	(0.0001)	(0.000)	(0.0001)
SD2 (ms)	0.843	0.889	0.892	0.991	0.837	0.993	0.610	0.793
	(0.014)	(0.006)	(0.003)	(0.0001)	(0.005)	(0.0001)	(0.014)	(0.004)

Data are reported as ICC (P value). HR_mean_: mean heart rate; RRi: RR intervals mean value; SDNN: RR intervals standard deviation; RMSSD: mean root square of differences between adjacent RRi divided by the number of RRi minus one; pNN50: percentage of differences between adjacent NN intervals that are greater than 50 ms; SD1: standard deviation type I; SD2: standard deviation type II; 1-RM: 1-repetition maximum test.

Bland-Altman plots of the differences between RMSSD during 3- and 2-min signals, RMSSD during 3- and 1-min signals, SD1 during 3- and 2-min signals, and SD1 during 3- and 1-min signals are reported in Figures 2 to [Fig f03] [Fig f04] 5, respectively. Results obtained for different resistance exercise loads (from 10% 1-RM to 35% 1-RM) are shown in panels A-D, respectively. The bias and the limits of agreement (1.96 SD of the bias) between values are indicated.

**Figure 2.** Bland-Altman plots of the differences between RMSSD during 3- and 2-min ignals at different resistance exercise loads. *A*, *B*, *C*, and *D* represent 10, 20, 30, and 35% 1-RM. The solid middle line indicates bias, while the two dashed lines represent the upper and lower limits of agreement. RMSSD: root mean square of the successive differences. 1-RM: 1-repetition maximum test.

**Figure 3. f03:** Bland-Altman plots of the differences between RMSSD during 3- and 1-min signals at different resistance exercise loads. *A*, *B*, *C*, and *D* represent 10, 20, 30, and 35% 1-RM. The solid middle line indicates the bias, while the two dashed lines represent the upper and lower limits of agreement. RMSSD: root mean square of the successive differences. 1-RM: 1-repetition maximum test.

**Figure 4. f04:** Bland-Altman plots of the differences between SD1 during 3- and 2-min signals at different resistance exercise loads. *A*, *B*, *C*, and *D* represent 10, 20, 30, and 35% 1-RM. The solid middle line indicates the bias, while the two dashed lines represent the upper and lower limits of agreement. SD1: short-term RRi standard deviation; 1-RM: 1-repetition maximum test.

**Figure 5.** Bland-Altman plots of the differences between SD1 during 3- and 1-min signals at different resistance exercise loads. *A*, B, C, and D represent 10, 20, 30, and 35% 1-RM. The solid middle line indicates the bias, while the two dashed lines represent the upper and lower limits of agreement. SD1: short-term RRi standard deviation; 1-RM: 1-repetition maximum test.

## Discussion

To our knowledge, this is the first study to investigate ultra-short-term HRV analysis during low-intensity resistance exercise, when signal stability is guaranteed. The main findings of this study are that no difference was found between HRV signals of different durations (1, 2, and 3 min) and that excellent to near-perfect association and good concordance were observed between parameters obtained from 1- and 2-min signal sections and from 3-min signal sections selected from 4-min signals recorded during the whole exercise session.

### Ultra-short-term HRV during resistance exercise

HRV measurements may help determine the timing of intensive training sessions based on the autonomic regulation status, even in the presence of declined, vaguely mediated beat-to-beat HRV (31 [Bibr B32]–33). Studies have demonstrated that it is possible to assess metabolic transition during dynamic resistance exercise in healthy elderly subjects by HRV indices calculation. Specifically, HRV indices are associated with blood-lactate levels, whose invasive measurement is the gold standard method to identify metabolic alterations during resistance exercise training (10,11). The exercise protocols used in these studies were limited to lower intensities (3 or 4 min of exercise), in order to guarantee the recording of stationary signals (1). Nevertheless, they analyzed exercises of around 48 repetitions, which is not recommended for clinical practice by the ACSM (14).

In order to improve the reliability of HRV monitoring during exercise, analysis methods that can be performed on short recordings are desirable, but currently lack investigation. In the present study, it was possible to verify that the analysis of 1- and 2-min stationary time series could provide a valid representation of physiological behavior, when a low-intensity resistance exercise is performed by elderly subjects. Thus, when approximately 20 exercise repetitions are performed, which is common in clinical practice, ultra-short-term HRV analysis appears feasible (14). Because resistance exercises for the elderly promote the gain of bone and muscle mass and the improvement of cardiovascular behavior, physical capacity, and quality of life, studies that assess HRV during experimental exercise programs appropriate for the training of this population are of great importance (34).

Studies have shown that ultra-short-term HRV analysis can be performed over 1-min signals recorded during rest in different populations and in different situations (15–23). Thong et al. (16) showed that time domain parameters (RRi and RMSSD) calculated over 1-min signals present high concordance with parameters calculated over 5-min signals in healthy adults. Furthermore, McNames and Aboy (17 [Bibr B18] [Bibr B19]) found that 1-min signals present good concordance with 5-min signals when RRi and RMSSD are compared in healthy adults.

Baek et al. (21) showed that some time and frequency domain indices, as well as some non-linear indices, can be calculated in physiology studies when ultra-short HRV segments are available. Munoz et al. (22) showed that it is unnecessary to use recordings longer than 120 s to obtain accurate measurements of RMSSD and SDNN in healthy adults. In diabetes patients, a study demonstrated that HRV indices can be reliably obtained from 1-min stationary signals (20).

Flatt and Esco (35) demonstrated that ultra-short-term HRV analysis can be performed during rest in the supine position in male and female university cross-country athletes, with near-perfect concordance between 1- and 10-min stationary signals for the natural log of RMSSD (LnRMSSD). These studies support ultra-short-term HRV analysis in physiological studies such as the one hereby presented.

Regarding exercise, some studies investigated ultra-short-term HRV during recovery. Esco and Flatt (23) observed that, after aerobic exercise, normalized LnRMSSD presented excellent concordance when 1- and 5-min time series were compared in athletes, when signal stability was guaranteed. In another study, Nakamura et al. (24) observed the same behavior for LnRMSSD in soccer players. These studies confirmed the possible use of ultra-short-term HRV analysis in young athletes. In the present study, ultra-short-term HRV was analyzed for the first time in different domains and during dynamic resistance exercise in healthy elderly individuals.

Currently, there is enormous interest towards studies that try to identify the beneficial effects of dynamic resistance exercise and criteria for safe prescription in the elderly, mainly due to the positive effects that this exercise modality induces (36,37). Therefore, a better understanding and precise characterization of the autonomic response during dynamic resistance exercise are of great importance in this population.

The high concordance observed between longer and shorter HRV signals in the present study may confirm the applicability of ultra-short-term HRV analysis in the time domain, as well as for the computation of non-linear indices, during low-intensity resistance exercise in the elderly, when signal stationarity is guaranteed. However, future studies are needed to confirm ultra-short-term HRV analysis reliability during resistance exercise when high intensities are applied.

### Limitations

The main limitation of the present study is that only healthy elderly men were tested, making it impossible to infer about the HRV behavior in female individuals or in patients affected by any kind of disease. The authors believe that considerable variability could be observed when analyzing these individuals. Moreover, it should be considered that the duration of each exercise session (4 min) was limited by the individuals' difficulty to perform resistance exercise for an extended period. Furthermore, it was impossible to assess ultra-short-term HRV at higher exercise intensities because signal stationarity could not be guaranteed while the subjects performed high-intensity resistance exercise. Future studies should focus on further refining HRV analysis by investigating: 1) cohorts with differing characteristics; 2) different exercise modalities and intensities; 3) different HRV signal durations.

Agreement was observed between 3-min stationary HRV signals and 1- and 2-min stationary HRV signals. Furthermore, concordance was observed between 3- and 1-min signals, which corresponds to the exercise duration prescribed in most dynamic resistance exercise programs applied in clinical practice. These findings suggest that, as long as signal stationarity is guaranteed, ultra-short-term HRV analysis in the time domain and in the non-linear domain could be applied as a more streamlined approach to HRV investigation.

## References

[1] Task Force of the European Society of Cardiology, the North American
Society for Pacing and Electrophysiology (1996). Heart rate variability - standards of measurement, physiological
interpretation, and clinical use. Circulation.

[2] Li HR, Lu TM, Cheng HM, Lu DY, Chiou CW, Chuang SY (2016). Additive value of heart rate variability in predicting
obstructive coronary artery disease beyond Framingham risk. Circulation J.

[3] De Bruyne MC, Kors JA, Hoes AW, Klootwijk P, Dekker JM, Hofman A (1999). Both decreased and increased heart rate variability on the
standard 10-s electrocardiogram predict cardiac mortality in the elderly The
Rotterdam Study. Am Heart J.

[4] Dekker JM, Schouten EG, Klootwijk P, Pool J, Swenne CA, Kromhout D (1997). Heart rate variability from short electrocardiographic recordings
predicts mortality from all causes in middle-aged and elderly men. The
Zutphen Study. Am J Epidemiol.

[5] Melo RC, Santos MD, Silva E, Quitério RJ, Moreno MA, Reis MS (2005). Effects of age and physical activity on the autonomic control of
heart rate in healthy men. Braz J Med Biol Res.

[B06] Kluttig A, Schumann B, Swenne CA, Kors JA, Kuss O, Schmidt H (2010). Association of health behaviour with heart rate variability: a
population-based study. BMC Cardiovasc Disord.

[B07] Melo RC, Takahashi ACM, Silva E, Martins LEB, Catai AM (2008). High eccentric strength training reduces the heart rate
variability in healthy older men. Br J Sports Med.

[8] Kiviniemi AM, Hautala AJ, Kinnunen H, Nissilä J, Virtanen P, Karjalainen J (2010). Daily exercise prescription on the basis of HR variability among
men and women. Med Sci Sports Exerc.

[9] Caruso FR, Arena R, Phillips SA, Bonjorno JC, Mendes RG, Arakelian VM (2015). Resistance exercise training improves heart rate variability and
muscle performance: a randomized controlled trial in coronary artery disease
patients. Eur J Phys Rehabil Med.

[10] Simões RP, Castello V, Mendes RG, Archiza B, Dos Santos DA, Bonjorno JC (2014). Identification of anaerobic threshold by analysis of heart rate
variability during discontinuous dynamic and resistance exercise protocols
in healthy older men. Clin Physiol Funct Imaging.

[11] Simões RP, Mendes RG, Castello V, Machado HG, Almeida LB, Baldissera V (2010). Heart-rate variability and blood-lactate threshold interaction
during progressive resistance exercise in healthy older men. J Strength Cond Res.

[B12] Machado HG, Simoes RP, Mendes RG, Castello V, Di Thommazo L, Almeida LB (2011). Cardiac autonomic modulation during progressive upper limb
exercise by patients with coronary artery disease. Braz J Med Biol Res.

[13] Machado-Vidotti HG, Mendes RG, Simões RP, Castello-Simões V, Catai AM, Borghi-Silva A (2014). Cardiac autonomic responses during upper versus lower limb
resistance exercise in healthy elderly men. Braz J Phys Ther.

[14] American College of Sports Medicine (2014). ACSM's Guidelines for exercise testing and prescription.

[15] Tulppo MP, Makikallio TF, Takala TES, Seppanen T, Huikuri HV (1996). Quantitative beat-to-beat analysis of heart rate dynamics during
exercise. Am J Physiol.

[16] Thong T, Li K, McNames J, Aboy M, Goldstein B (2003). Accuracy of ultra-short heart rate variability
measures. IEEE.

[17] McNames J, Aboy M (2006). Reliability and accuracy of heart rate variability metrics versus
ECG segment duration. Med Biol Eng Comput.

[B18] Salahuddin L, Cho J, Jeong MG, Kim D (2007). Ultra short term analysis of heart rate variability for
monitoring mental stress in mobile settings. IEEE.

[B19] Kiviniemi AM, Breskovic T, Uglesic L, Kuch B, Maslov PZ, Sieber A (2012). Heart rate variability during static and dynamic breath-hold
dives in elite divers. Auton Neurosci.

[20] Nussinovitch U, Cohen O, Kaminer K, Ilani J, Nussinovitch N (2012). Evaluating reliability of ultra-short ECG indices of heart rate
variability in diabetes mellitus patients. J Diabetes Complic.

[21] Baek HJ, Cho CH, Cho J, Woo JM (2015). Reliability of Ultra-short-term analysis as a surrogate of
standard 5-min analysis of heart rate variability. Telemed J E-Health.

[22] Munoz ML, van Roon A, Riese H, Thio C, Oostenbroek E, Westrik I, Geus et al (2015). Validity of (Ultra) short recordings for heart rate variability
measurements. PLoS One.

[23] Esco MR, Flatt AA (2014). Ultra-short-term heart rate variability indexes at rest and
post-exercise in athletes: evaluating the agreement with accepted
recommendations.

[24] Nakamura FY, Flatt AA, Pereira LA, Ramirez-Campillo R, Loturco I, Esco MR (2015). Ultra short-term heart rate variability is sensitive to training
effects in team sports players. J Sports Sci Med.

[25] American College of Sports Medicine (2002). Position stand on the appropriate intervention strategies for
weight loss and prevention of weight regain for adults. Med Sci Sports Exerc.

[26] Balady GJ, Chaitman B, Driscoll D, Foster C, Froelicher E, Gordon N (1998). Recommendations for cardiovascular screening, staffing, and
emergency policies at health/fitness facilities. AHA/ACSM Scientific
Statement. Circulation.

[27] American College of Sports Medicine (2002). Position stand on the appropriate intervention strategies for
weight loss and prevention of weight regain for adults. Med Sci Sports Exerc.

[28] Borg GA (1982). Psychophysical bases of perceived exertion. Med Sci Sports Exerc.

[29] Mourot L, Bouhaddi M, Perrey S, Rouillon JD, Regnard J (2004). Quantitative Poincaré plot analysis of heart variability: effect
of endurance training. Eur J Appl Physiol.

[30] Hopkins WG (2002). A Scale of magnitudes for effect statistics. A New view of statistics.

[31] Plews DJ, Laursen PB, Kilding AE, Buchheit M (2012). Heart rate variability in elite triathletes, is variation in
variability the key to effective training? A case comparison. Eur J Appl Physiol.

[B32] Plews DJ, Laursen PB, Stanley J, Kilding AE, Buchheit M (2013). Training adaptation and heart rate variability in elite endurance
athletes: opening the door to effective monitoring. Sports Med.

[33] Da Silva DF, Verri SM, Nakamura FY, Machado FA (2014). Longitudinal changes in cardiac autonomic function and aerobic
fitness indices in endurance runners: A case study with a high-level
team. Eur J Sport Sci.

[34] Csapo R, Aledre LM (2016). Effects of resistance training with moderate *vs*
heavy loads on muscle mass and strength in the elderly: A
meta-analysis. Scand J Med Sci Sports.

[35] Flatt AA, Esco MR (2016). Evaluating Individual training adaptation with smartphone-derived
heart rate variability in a collegiate female soccer team. J Strength Cond Res.

[36] Peterson MD, Sen A, Gordon PM (2011). Influence of resistance exercise on lean body mass in aging
adults: a meta-analysis. Med Sci Sports Exerc.

[37] Dias CP, Toscan R, de Camargo M, Pereira EP, Griebler N, Baroni BM (2015). Effects of eccentric-focused and conventional resistance training
on strength and functional capacity of older adults. AGE.

